# Presentation of Novel Hybrid Algorithm for Detection and Classification of Breast Cancer Using Growth Region Method and Probabilistic Neural Network

**DOI:** 10.1155/2021/5863496

**Published:** 2021-06-19

**Authors:** Zeynab Nasr Isfahani, Iman Jannat-Dastjerdi, Fatemeh Eskandari, Saeid Jafarzadeh Ghoushchi, Yaghoub Pourasad

**Affiliations:** ^1^Ahvaz Jundishapur University of Medical Sciences, Ahvaz, Iran; ^2^Department of Radiology, School of Medicine, Isfahan University of Medical Sciences, Isfahan, Iran; ^3^Department of Industrial Engineering, Urmia University of Technology, Urmia, Iran; ^4^Department of Electrical Engineering, Urmia University of Technology, Urmia, Iran

## Abstract

Mammography is a significant screening test for early detection of breast cancer, which increases the patient's chances of complete recovery. In this paper, a clustering method is presented for the detection of breast cancer tumor locations and areas. To implement the clustering method, we used the growth region approach. This method detects similar pixels nearby. To find the best initial point for detection, it is essential to remove human interaction in clustering. Therefore, in this paper, the FCM-GA algorithm is used to find the best point for starting growth. Their results are compared with the manual selection method and Gaussian Mixture Model method for verification. The classification is performed to diagnose breast cancer type in two primary datasets of MIAS and BI-RADS using features of GLCM and probabilistic neural network (PNN). Results of clustering show that the presented FCM-GA method outperforms other methods. Moreover, the accuracy of the clustering method for FCM-GA is 94%, as the best approach used in this paper. Furthermore, the result shows that the PNN methods have high accuracy and sensitivity with the MIAS dataset.

## 1. Introduction

Breast cancer is a deadly and frequent illness that affects people all over the world. In the next 20 years, the number of new breast cancer patients is expected to increase by 75 percent. Consequently, according to the WHO in 2019, precise and early detection plays a critical role in developing the diagnostic and increasing the patients' survival rate with breast cancer from 20% to 60%. Tumors come in various forms that must be identified independently since each might lead to different treatment options and prognoses [1]. To aid oncologic decision-making, cancer categorization strives to give an accurate diagnosis of the illness and a prognosis of tumor activity. Traditional breast cancer categorization, which is mainly focused on clinicopathologic aspects and the use of routine biomarkers, may not represent the wide range of clinical outcomes experienced by individual breast cancers. The biology that underpins cancer genesis and progression is complex. Recent high-throughput technology results have added to our understanding of breast cancer's underlying genetic changes and biological processes [2].

Mammography is the most effective method for the early detection of breast cancer [3]. However, a look back reveals that many lesions that can be seen on a mammogram are overlooked by radiologists, which can have various causes, such as poor quality of the mammogram image, benign appearance of the lesions, and eye fatigue or neglect by radiologists. Utilizing diagnostic approaches in the early stages of cancer development can be very effective and essential for patient treatment so that this early diagnosis can help doctors treat patients and significantly reduce the mortality of patients. Examination of breast tumors has a special place in the initial diagnosis of breast cancer [4]. Due to this, diagnosis with the eye can be prone to error, and the radiologist may not identify the tumor and cancer. Therefore, having an image processing system with the power to extract features that the human eye cannot detect or recognize with low accuracy can be very useful. A tumor is an abnormal mass of cells. Tumor cells grow for reasons that are still unknown, and they grow regardless of the body's needs [5]. Moreover, because nutrients absorb normal cells from the blood, they are often harmful to the body. Tumors are often called neoplasms or neoplasms. Body tissues are permanently repaired and replaced with new cells following damage or damage caused by natural cell depletion. Therefore, in general, growth and repair depend on the body's needs. Specific organs can grow in size (hypertrophy) or increase the number of cells (hyperplasia) if the organ is required to do more than its capacity [6].

A breast cancer diagnosis can help physicians to treat patients and significantly reduce mortality. Also, it increases the 5-year survival rate of patients with this cancer from 14% to 49% [7]. It is very important to check for breast cancer and to diagnose the tumor quickly and accurately. It is because eye diagnosis can be prone to error, and the radiologist may not detect the tumor. Therefore, there is an image processing system with high extraction power for detecting tumors, which can be very useful. The reduction in breast cancer mortality during screening may be even more significant. Since investigations have revealed that radiologists have failed to identify a remarkable number of breast cancer cases, the reasons for these cases are the failure of mammography screening. It is often unclear that disorders that are not visible in the images should be ignored. However, cancer may not be detected due to the absence of symptoms. Computer-aided diagnosis (CAD) is being developed. These methods utilized pattern recognition approaches to find features in the image that characterize breast cancer tumor location. Therefore, CAD systems assist the radiologist during the examination [8]. The image of suspicious areas is used. Most CAD systems also have diagnostic errors. However, there is also evidence that the CAD system can enhance the radiologist's ability to interpret detection lesions. Although the results of a small number of recent studies indicate that the performance of existing commercial CAD systems still needs to be developed, they can meet the needs of imaging centers and clinics. Therefore, improving the performance of CAD systems is a crucial issue for investigation, and future developments remain [9].

The convolutional neural network (CNN) is a multilayer system that recovers features from raw input. It is a symbol for hierarchical structuring [10]. Convolution layers, fully connected layers, pooling, and an output layer are among the layers that make up a deep neural network (DNN) [11]. A convolution layer is one of these layers that is beneficial for learning high-level characteristics such as the edges of an image. FC layers are used to learn pixel-by-pixel characteristics. A pooling layer can minimize the quantity of convolved features, lowering the amount of computing power required. Max pooling and average pooling are two operations that this layer may execute [12, 13]. There are two types of CNNs utilized for breast image or data classification: de novo trained models and transfer learning-based models. The term “de novo model” refers to CNN-based models created and trained from the ground up [14]. On the contrary, transfer learning networks are CNN models that use previously trained neural network models such as AlexNet, visual geometry group, and residual neural network [15, 16].

This study aims to cluster the breast cancer area using the region growth method in combination with the FCM-GA approach. These results are compared with the manual selection method and Gaussian Mixture Model method for verification. In the second part of the paper, the classification is performed to diagnose breast cancer type in two datasets of MIAS and BI-RADS using features of GLCM and probabilistic neural network (PNN).

## 2. Literature Review

Veena and Padma [17] preprocessed the input image by reducing the noise coefficient using the intermediate filter method, reducing the image noise. Then, they use Gaussian mixed model (GMM), one of the well-known clustering algorithms for image segmentation, and finally, by applying probabilistic neural network (PNN) classifier on the features extracted with coincident matrix algorithm. Gray area (GLCM) is classified into three categories of benign, malignant, and normal cases. Punitha et al. [18] used intelligent artificial bee colonization and Improved Monarch Butterfly Optimization Technique (IABC-EMBOT) to detect breast cancer. The method used is of good speed and accuracy. Classification accuracy is 97.53%, sensitivity is up to 96.75%, specificity is up to 97.04%, and the average processing time is 113.42. Sakri et al. [19] presented a feature selection method for predicting the recurrence of breast cancer. The selection method is the Particle Swarm Optimization (PSO-RM) feature which uses three different classifiers KNN, NB, and the fast decision tree. Among the 34 features, the proposed method chooses the best quadratic method and improves the accuracy of all three classifiers. KNN accuracy improved from 70% to 81%, NB from 76% to 80%, and the fast decision tree from 66% to 75%.

Karthik et al. [20] used a deep neural network to learn data characteristics (DNNs). They categorized breast cancer data using multiple-layer DNNs. Experimental results show that the accuracy obtained from this system is 97.66%, and the sensitivity is slightly less than 0.98. The deep network designed in this study is for breast cancer datasets only. Unni et al. [21] used a general thresholding method to estimate the basal chest muscle boundary and then applied morphological methods to correct the extracted area boundaries and the mean filter to eliminate noise. The GLCM algorithm is used to extract the property. Then, a subset of these features that provides the best classification rate is selected using a genetic algorithm. Finally, Support Vector Machine Classification (SVM) is used to classify benign and malignant cancers.

Selvathi and Poornila [22] propose a general thresholding method for extracting chest bounds in images in which images are converted to binary using a fixed threshold value of 18. Each component with a significant number of pixels connected is considered as the chest area. The region boundary is then smoothed using a disk with a radius of 5 pixels using morphologically based filtering operations. Sasikala and Ezhilarasi [23] also proposed a general thresholding method for the extraction of breast boundaries. The 8-bit image noise used by the mean filter is reduced, and the image contrast is improved by the Contrast Limited Adaptive Histogram Equalization (CLAHE) algorithm. The images are then converted to binary images with a fixed threshold value followed by morphology-based filtering operations to eliminate small background objects. Results reported for this study included a maximum accuracy of 97.1%, a sensitivity of 98.8%, and a specificity of 95.4%. Heidari et al. [24] took mammographic image features and created an optimal classification model to estimate the risk of breast cancer. The data analyzed are 500 and divided into 50% high risk and 50% low risk. To anticipate the risk of cancer diagnosis, they proposed an LPP model based on the combination of several features to reduce the dimensions of the feature space. Unlike typical feature selection techniques that select a set of optimal features from the primary feature, LPP creates a new optimum feature array that includes features different from the main features in the feature pool, which ultimately created a 9.7% rise in risk anticipation accuracy.

Tariq et al. [25] conducted a study to classify mammographic images of breast cancer. GLCM algorithm was used to extract texture-type features from images. Then, a smaller set was made by the individual, in addition to the whole set of features. 60% of the data is used for training, 20% for validation, and 20% for testing. Using ANN as a classifier, the results of this study achieved 99% accuracy in the image recognition process. Kashyap et al. [26] used a partial differential equation adjustment process to extract the chest area, mammogram images, dark masking, and moderate filtering and map suspicious anomalies. Fuzzy c-mean clustering is applied. To calculate the texture characteristics of suspected fragmented masses, the local binary pattern was rotated, and local binary patterns were calculated. At the end of the support vector machine, polynomial kernel and radial basis function and multilayer and linear perceptron were used to classify areas of suspicion of abnormal and ordinary clades.

Chowdhary et al. [43] used the fuzzy c-mean bounded probability (IPFCM) method to overcome the bugs in traditional methods, namely, noise and random clustering, and used a fuzzy histogram algorithm in initial preprocessing in mammographic images. Finally, extraction, classification, and validation are performed to assist the radiologist in tumor diagnosis.

Rampun et al. [44] used a pretrained modified version of AlexNet with detailed adjustments in the database of CBIS-DDSM mammography images. The AlexNet network architecture used different parameters with more advanced functions such as PReLu instead of ReLu. The experimental results of this study are classification accuracy (ACC) of 80.4% and area under the curve (AUC) of 0.84. Kim et al. [45] evaluated the feasibility of using data-driven imaging biomarkers (DIB-MG) to characterize the deep CNN algorithm in mammographic images, including normal and benign classes. Using the algorithm, they have achieved a sensitivity of 76% and a specificity of 89%.

Zhang et al. [46] used a neural network algorithm to classify mammographic images. They evaluated ten different CNN architectures and concluded that combining both data addition methods (each original image into eight images) and a circular neural network would improve classification performance. The area under the ROC curve is 0.73. Salama et al. [47] developed a new computer-aided diagnosis (CAD) system to diagnose breast cancer in digital mammography. They used the WBCT algorithm to extract the feature. GA-SVM-MI optimization technique was used to select the optimal set of features. In this algorithm, the classification accuracy is between normal-abnormal (97.5%) and benign (96%) cases (see Table 1).

## 3. Methods and Materials

### 3.1. Data Collection

MIAS (Mammography Image Analysis Society), a UK research community engaged in understanding mammography, is a database for digital mammograms that have been developed. Films taken from the UK National Breast Screening Program were digitized with a Joyce-Loebl scanning microdensitometer to the 50-micron pixel tip, a linear unit in the optical density range 0–3.2, and an 8 bit term for each pixel. The list is split into film pairs, where each pair reflects a single patient's left (even filename numbers) and right (odd filename numbers) mammograms. The file resolution is 1024 pixels x 1024 pixels for ALL images. In the matrix, the images have been centered. Center positions and radii, rather than individual calcification, refer to clusters when calcification is present. The bottom-left corner is the root of the coordination system. In some cases, calcification is widely dispersed rather than concentrated at a single position throughout the image. Center positions and radii are unsuitable in these situations and removed [48].

The second dataset is a BI-RADS data collection intended to standardize reporting on breast imaging and minimize uncertainty in the understanding of breast imaging. It also promotes monitoring of outcomes and evaluation of quality. It provides a lexicon for systematic terminology and chapters on report organizations and guidance for use in everyday practice, for Mammograms, US breast, and MRI. A database of clinical mammograms comprising 60 patient photos was taken from mammogram screening centers. A broad range of cases that are difficult to classify by radiologists is included in the real-time database. Both clinical mammograms obtained from screening clinics were positive for abnormalities in their presence. Initially, as an input, we take a 2D mammogram image of size M×N and add the average filter to it. The pictures are 20 benign, 20 malignant, and 20 regular images of the breast tumor.

### 3.2. Growth Region Algorithm

This approach focuses on the definition employed to divide the image into distinctive regions to analyze the homogeneity and centered on the resemblance or the homogeneity of the neighboring pixels. The pixels in each region are comparable to particular parameters, such as color and strength. These histogram-based image clustering approaches concentrate only on the dispersion of image pixels at the grayscale, whereas district growth techniques note that near-gray levels are often present in the surrounding pixels.

Area-based methods are performed as follows:

1. The beginning of the algorithm is regarded to be the number of initial seeds.
2. The region starts to develop from these seeds. The pixels are inserted in this area similar to the initial pixels.
3. The next grain is considered when the region's growth ends, and the following area's growth continues.
4. These steps keep going until one region belongs to all the pixels in the image.

The following measures refer to the growth method of the region (Figure 1).

Step 1: *select initial seeds*. It must manually insert the initial points to start the algorithm. In the handy process, the algorithm begins by choosing the initial points for the user. Several techniques automatically take out the initial points in the sector: the utilization of a random step algorithm to identify the first points, for instance. To pick the initial points, this study proposes an algorithm that focuses on FCM-GA methods. The purpose of the algorithm is to use the fuzzy clustering algorithm to implement clustering initially. Moreover, it is distinguished by membership grade *M* and cluster centers *C*. Then, through the genetic algorithm, the appropriate values of these parameters are gained based on reducing target function. In the following approach, the error performance criterion *E* is

(1) $$\begin{array}{c} E\left(C\right)=\sum_{j=1}^{n}\overset{K}{\underset{i=1}{\sum }}m_{ij}x_{j}-c_{iA}^{2}, \end{array}$$

where the *m* relation is as follows:

(2) $$\begin{array}{c} 0<\overset{n}{\underset{j=1}{\sum }}m_{ij}<n,\;\;i=1,2,\ldots ,K,\\ \overset{K}{\underset{i=1}{\sum }}m_{ij}=1,\;j=1,2,\ldots ,n,\\ \overset{K}{\underset{i=1}{\sum }}\overset{n}{\underset{j=1}{\sum }}m_{ij}=n. \end{array}$$

Furthermore, from the following relationship, *m* and *C* are computed:

(3) $$\begin{array}{c} m_{ij}={\left[\sum_{k=1}^{K}\left(\frac{x_{j}-c_{iA}}{x_{k}-c_{i}}\right)\sum \right]}^{-1},\;1\leq i\leq K\;,\;1\leq j\leq n,\\ c_{i}=\frac{\sum_{j=1}^{n}m_{ij}x_{j}}{\sum_{j=1}^{n}m_{ij}},\;1\leq i\leq K. \end{array}$$

Step 2: *determine the similarity of regions*. The selection of the similarity criterion between the regions is achieved. Then, the initial points have been defined in the previous stage. The criterion of similarity is utilized to evaluate the resemblance of the new pixels. The pixels of the regions define the assignment of the new pixel to the corresponding area.

The standard deviation criterion is one of these criteria for similarity. The new pixel *I*_*n*+1_(*x*, *y*) relates to the region when it is used under the following condition and is used in the mean and standard deviation areas:

(4) $$\begin{array}{c} \mu_{n}-X\sigma_{n}\;<I_{n+1}\left(x+y\right)<\mu_{n}+X\sigma_{n}, \end{array}$$

where *X* is a variable that describes the difference in the area by how many pixels, usually, 99.7% of the actual seeds in the field, are placed in an isolated area where *X* is considered to be 3. The smaller *X* is, the fewer points the region contains, and the picture splits into more regions. The threshold criterion is another deemed criterion. In this process, the average of the regions is determined, and the new pixel *I*_*n*+1_(*x*, *y*) relates to the area as the following condition:

(5) $$\begin{array}{c} \mu_{n}-X<I_{n+1}\left(x+y\right)<\mu_{n}+X. \end{array}$$

In this context, when the gap is less than the defined limit between the pixels and the average area, the area covers that pixel. For color images (red, green, and blue), this situation must also extend to all three layers to connect these pixels to this region.

Step 3: *the third step is growth region*. The region's growth is carried out after choosing the initial seeds for beginning the algorithm and the criterion of similarity for pixels with zones. The area's development is such that the adjacent regions are chosen, beginning from the initial seeds.

### 3.3. Fuzzy C-Means (FCM)

FCM Bezdek et al. (1984) developed a classification algorithm regarding the reductions of the objective function:

(6) $$\begin{array}{c} J_{q}=\sum_{i=1}^{n}\sum_{j=1}^{m}u_{ij}^{q}d\left(x_{i},\theta_{j}\right), \end{array}$$

where *q* manages the nonresolution degree and the classification spike.

U seems to be the inextensible membership in the center class of the *x*_*i*_ data. The interval between the *x*_*i*_ data and the middle of class *j* and *d* should be the interval.

U is subject to the following situations:

(7) $$\begin{array}{c} u_{ij}\in \left[0,1\right],\overset{n}{\underset{j=1}{\sum }}u_{ij}=1\&0<\overset{n}{\underset{j=1}{\sum }}u_{ij}<n. \end{array}$$

For each group of the following relationships, the membership function and center membership are gained:

(8) $$\begin{array}{c} u_{ij}=\frac{1}{{}_{\sum }^{m}{\left(d\left(x_{i},\theta_{j}\right)/d{\left(x_{i,}\theta \right)}_{i}\right)}^{2/\left(q-1\right)}},\\ \theta_{j}=\frac{\sum_{k=1}^{N}u_{ij}^{q}x_{i}}{\sum_{k=1}^{N}u_{ij}^{q}}, \end{array}$$

### 3.4. Genetic Algorithm (GA)

The genetic algorithm (GA) is an optimization tool based on the Darwinian evolutionary rule. In each step of applying the GA, a set of search points is applied to arbitrary processing. Every point has appointed a sequence of characters in this method, and genetic operators carry out these sequences. To obtain new results in the search space, the resulting sequences are then diced. In the end, the likelihood of their presence in the next level is calculated based on the premise that each point has an objective function.

The fitness function was described in this research as follows. This function is determined based on the difference between the degraded database image and the image acquired by the growth method of the field, beginning at the initial random point, as follows:

(9) $$\begin{array}{c} \text{cost}={\left(G-I_{1}\right)}^{2}+{\left(W-I_{2}\right)}^{2}+{\left(B-I_{3}\right)}^{2}, \end{array}$$

where gray, white, and black layers are  *I*_1_ and *I*_3_ are images derived from fragmentation, respectively.

### 3.5. Adaptive Median Filter

The adaptive median filter classifies each pixel of the image as noise with its surrounding pixels. The size of the neighborhood, as well as the reference threshold, are adjustable. As impulse noise, a pixel that varies from most of its neighbors and is not functionally compatible with those pixels to which it is identical is labeled. The objects are (1) deleteing noise from impulse, (2) smoothing other noises, and (3) diminishing distortion, such as extreme thinning or object boundary thickening [49].

### 3.6. Gaussian Mixture Model

As a random parameter, the pixel's value in an image (i.e., the intensity or color) can be taken. Since each random variable has a probability distribution, then pixel values have a distribution of probability [50]. A reasonable probability distribution for pixel values of an image is the Gaussian mixture distribution. The form is the Gaussian mixture distribution formula:

(10) $$\begin{array}{c} f\left(x_{s}\right)=\sum_{i=1}^{k}P_{i}N\left(x_{s}|\mu_{i},\sigma_{i}\right), \end{array}$$

where

(11) $$\begin{array}{c} N\left(x_{s}|\mu_{i},\sigma_{i}\right)=\frac{1}{\sigma_{i}\sqrt{2\pi }}\exp\left[-\frac{1}{2\sigma_{i}^{2}}{\left(x_{s}-\mu_{i}\right)}^{2}\right]. \end{array}$$

We presume that an image is categorized into a *C*_*i*_=1,2,…,  *k* class known to the class *k*.  *μ*_*i*_, *σ*_*i*_^2^, and *p*_*i*_ parameters are of *C*_*i*_-class in terms of mean, variance, and likelihood.

It means the following:

(12) $$\begin{array}{c} p_{i}=p\left(x_{s}\in C_{i}\right),\;0<p_{i}<1,\\ \;\overset{k}{\underset{i=1}{\sum }}p_{i}=1. \end{array}$$

### 3.7. Expectation-Maximization Algorithm

In setup to the K-means, the EM algorithm is very identical. Similarly, choosing the input partitions is the first part. In this case, to compare findings more realistic, the same initial partitions as utilized in the color segmentation with K-Means were used. Here is the comparison parameter, RGB color was again chosen. The EM cycle starts with the following equation described by an Expectation phase [51]:

(13) $$\begin{array}{c} E\left[z_{ij}\right]=\frac{p\left(x_{i}|\mu_{i}\right)}{\sum_{n=1}^{k}p\left(x_{i}|\mu_{i}\right)}=\frac{\exp\left[-1/2\sigma_{i}^{2}{\left(x_{s}-\mu_{i}\right)}^{2}\right]}{\sum_{n=1}^{k}\exp\left[-1/2\sigma_{i}^{2}{\left(x_{s}-\mu_{i}\right)}^{2}\right]}. \end{array}$$

This equation asserts that concerning partition *j*, the assumptions or weight for pixel *z* equals the possibility that *x* is pixel *x*_i_ provided that *μ* is partition µ_i_ divided by the sum over all components *k* of the same probability subsequently defined. For weights, this contributes to the lower expression. The sigma expresses the covariance of pixel data squared shown in the second expression. The *M* step or maximization step starts once the *E* step has been implemented, and every pixel has a weight of expectation for each partition. The following equation defines this step:

(14) $$\begin{array}{c} \mu_{j}\leftarrow \frac{1}{m}\sum_{i=1}^{m}E\left[z_{ij}\right]x_{i}. \end{array}$$

This equation indicates that the partition value *j* is modified to the weighted average of the pixel values for this specific partition, where the weights are the weights of the *E* phase. For each new set of partitions, this EM loop is replicated until, as in the K-Means algorithm, the partition values do not shift by a significant amount anymore.

### 3.8. Hidden Markov Random Field Model (HMRFM)

HMRFM is defined by a sequence of observations as accidental processes generated by a sequence of Markov whose state sequence cannot be explicitly tracked. Each observation of the state series is presumed to be a stochastic function. According to the *l* × *l* transition probability matrix, in which *l* represents the number of states, the underlying Markov chain alters its state. HMMs have been effectively used in speech recognition and handwritten script recognition [52]. Since the original HMMs were created as 1D Markov chains, 2D/3D problems like image segmentation cannot be used directly with first-order neighborhood structures. Here, we consider an HMM case that contains a Markov random field rather than a Markov chain and thus is not confined to 1D as the underlying stochastic process. We call this particular case an HMRF model. The following characterizes an HMRF model mathematically:

- *Hidden Random Field (MRF).* Let *ℓ* be a finite status space with the distribution of probability; the arbitrary vector  *x*={*x*_*i*_ *i* ∈ *s*} is an underlying MRF (5). The condition of *X* is not observable.
- *Objective Random Field.y*={*y*_*i*_, *i* ∈ *s*} is a random field with space *D* as a finite state. Each *Y*_*i*_ is the conditional probability distribution *p* (*y*_*i*_ | *x*_*i*_) for function *f*(*y*_*i*_; *θ*_*xi*_) given any unique configuration*x* ∈ *X*, where the parameters associated are*θ*_*xi*_. The emission likelihood function is termed this distribution, and Y is often pointed to as the arbitrary vector released.
- *Conditional Dependency.* For any *x* ∈ *X*, the arbitrary parameters *Y*_*i*_ are conditional independent:

(15) $$\begin{array}{c} P\left(Y-X\right)={\prod^{}}_{i\in s}p\left(y_{i}|x_{i}\right). \end{array}$$

### 3.9. Probabilistic Neural Network (PNN)

The PNN is a network for neural feed-forward, widely employed in diagnosis and pattern recognition algorithm. According to the discriminant analysis of the Kernel Fisher, this form of ANN was extracted. The operations are categorized into four layers of a multilayered feed-forward network within a PNN as input, pattern, summation, and output layers (see Figure 2).

In classification problems, PNN is also utilized [53]. The first layer measures the difference when input is available, from the input vector to the training input vectors. The pattern layer calculates the relationship between each type of inputs and produces the net output as a likelihood vector. Eventually, a competitive transfer feature on the output of the second layer chooses the sum of those possibilities. For that class and nontarget classes, binary identification is created, respectively. Each neuron in the input layer defines a predictor variable. In categorical variables, when there are N category numbers, N-1 neurons are considered. The pattern layer includes a neuron for every case in the training process. It keeps the values of the input variables for the scenario, along with the output value. In the summation layer, the values for the class they represent are added by the pattern neurons. In the output layer, for each target category, it contrasts the weighted collected in the pattern layer and uses the maximum values to predict the targets.

### 3.10. ROC Curve

To determine the outcome of binary classification (duality), sensitivity and specificity are used in the statistics of both measures. The consistency of the outcomes of a test that separates the information into these two categories is observable and descriptive using sensitivity and attribute metrics when the data can be separated into positive and negative classes. Sensitivity means the percentage of positive cases that would be correctly checked as positive. Specificity means the percentage of negative cases that correctly label them as negative. The sensitivity is the division of true-positive cases in statistical terms into the sum of true-positive cases and false-negative cases:

(16) $$\begin{array}{c} \text{Sensitivity or recall}=\frac{\text{TP}}{\text{TP}+\text{FN}},\\ \text{Specificity}=\frac{\text{TN}}{\text{TN}+\text{FP}}. \end{array}$$

The sensitivity of the test and its specificity depend on the quality of the test and the type of test utilized. However, it is not possible to describe the outcome of a test using sensitivity and specificity alone:

(17) $$\begin{array}{c} \text{Precision}=\frac{\text{TP}}{\text{TP}+\text{FP}},\\ \text{Accuracy}=\frac{\text{TP}+\text{TN}}{\text{TP}+\text{TN}+\text{FP}+\text{FN}},\\ \text{Fall}-\text{out}=\frac{\text{FP}}{\text{FP}+\text{FN}}. \end{array}$$

The ROC curve is a plot displaying the diagnostic capabilities of the binary classifier system as its discrimination threshold is different. The ROC curve is formed by plotting the true-positive rate against fall-out or the false-positive rate at different threshold settings. Sensitivity, recall, or likelihood of identification are also recognized as the true-positive rate. Accuracy, specificity, and precision are other performance analysis parameters.

## 4. Results and Discussion

### 4.1. Presented Approach

The diagram of the approach presented is shown in Figure 3. We used the growth region technique for tumor detection and adaptive median filters for classification to eliminate noise from the image since it is best for all spatial filtering and recognizes noise from fine information. The Adaptive Median Filter implies space processing to evaluate the impulse noise pixels in an image. By comparing each pixel with its surrounding pixels in the image, the adaptive media filters classify pixels as noise. The size of the neighborhood, as well as the comparison threshold, is adjustable.

### 4.2. The Tumor Detection Stage

#### 4.2.1. Growth Region Method

In the growth region algorithm, the average value of the initial seeds is the average of the tumor area in this work, and the initial STD is equal by zero for region growth beginning from the initial seeds in the input image. Neighborhoods are referred to for their initial point 8. The analysis is done so that the pixels around it are checked, starting with the initial seed, and if they relate to that class, they are attached to it.

By accumulating points to that class as follows, the average and STD of the old class are recursively updated by using the mean and STD of the previous stage:

(18) $$\begin{array}{c} \mu_{N}=\frac{\left(N-1\right)\left(\mu_{N-1}\right)+I_{N}}{N},\\ \sigma_{N}=\sqrt{\frac{\left(N-2\right){\left(\sigma_{N-1}\right)}^{2}+N/N-1{\left(I_{N}-\mu_{N}\right)}^{2}}{N-1}}. \end{array}$$

Then, they will also be located in the same neighborhood, and the criteria for the neighboring point applied to this class will be changed. This search will continue until ultimately detecting the first class and not add any other point. The cluster size of the FCM is ten, and the population size of GA is 100. Furthermore, 0.2 is the rate of mutations.  Figure 4 shows the clustering findings using the FCM-GA approach mentioned. The precise location of the target tumor area was detected in the final image (see Figure 5).

#### 4.2.2. Segmentation Using GMM

The outcomes of Adaptive Median Filtration are also shown in Figure 6. The image is clarified, and the noise is reduced. These noise pixels would then substitute the value of the median pixel in the adjacency. Initially, the image is transformed into a grayscale image, adaptive median filtering is then applied to the output image, and the image is transformed to an integer eight that is unsigned. Then, with two regions, two GMM components, and 100 iterations, the GMM clustering is performed on the preprocessed image.

We used the k-means clustering method (*k* = 2) and applied HMRF-EM. Figures 7 and 8 display the effects of the GMM process. Malignant and benign tumors are illustrated in Figures 7 and 8, respectively, and we can segment the tumors using the presented procedure.

Figure 9 demonstrates the effects of the approach provided for normal breasts. The results do not reveal the critical section of the tumor in the model. Also, the chest muscle is present in the white position in the top corner of the figure.

#### 4.2.3. The Performances of Approaches

Table 2 shows the fuzzy fitness value with three presented techniques in the genetic algorithm and is compared by the maximum values of Jaccard and the minimum Jaccard distance. In the genetic algorithm, the FCM based fitness function works well due to similarities between the techniques and the smallest Jaccard distance.

The clustering methods are presented based on the growth region method. Then, the analysis was used in this work on a variety of performance criteria. The suggested approach can diminish the RMS error, as shown from the results (Table 3). It indicates that the division of the picture was performed more precisely. In this analysis, FCM-GA was employed to separate the initial points using the area growth process. As mentioned, the appropriate initial points have been selected using a genetic algorithm and evaluating the proper fitness function for image clustering using fuzzy logic. With this hybrid method, we get the required initial seeds for starting the growth process.

Consequently, the presented method was implemented on mammography MRI breast cancer images, and the outcomes were recorded. The finding revealed that the suggested algorithm could reduce the clustering error. We utilized 212 healthy breasts and 110 breast cancer images for the implementation of the algorithm. The performance criteria are shown in Table 4. The findings indicate that for presented techniques, maximum sensitivity is shown. Besides, the GMM approach offers minimal fall-out and optimum sensitivity with better detection performance using the GA to collect initial seeds.

We demonstrate that this method is appropriate according to the receiver operating characteristic (ROC) curve. Since it has a sensitivity above the line of guess, the optimal outcome should have minimal fall-out and optimum sensitivity concerning Figure 10.

### 4.3. The Classification Stages

We used two BI-RADS and MIAS datasets in the classification stage. We utilized 60 breast cancer images in BI-RADS, including 100 malignant and 100 benign breast cancer images.  Table 5 displays the sensitivity, fall-out, precision, accuracy, and specificity parameters of classification using the PNN method. The result shows that the PNN methods have high accuracy and sensitivity with the MIAS dataset. Also, the fall-out for the MIAS dataset is 0.08, which is lower than BI-RADS as 0.8, so the number of datasets will trigger classification outcomes.

## 5. Conclusion

In this study, an automated clustering method is proposed to detect breast cancer from mammographic MRI images based on the growth region method. Also, FCM-GA was utilized to find initial seeds. MRI images are proposed for target area detection and extraction utilizing genetic algorithm-based dynamic image analysis. Comparison results of RMSE error reveal that the suggested algorithm has the lowest error rates relative to the other method. Moreover, the suggested FCM-GA method has a higher Jaccard index and the minimum Jaccard distance than other methods.

Moreover, the suggested GMM solution is close to the method of FCM-GA. As shown in the findings, the RMS error could be minimized by the suggested approach. For the automatic selection of the appropriate initial seeds, a genetic algorithm has been used based on fuzzy logic clustering techniques to start the growth process. Also, we used the adaptive median filter for classification to eliminate noise from the picture of breast cancer, to distinguish between fine details and noise. We then performed the GMM clustering on the preprocessed image. Moreover, the PNN method is used to classify or diagnose tumor types based on GLCM features extracted from GMM resulted in images. We utilized two datasets MIAS and BI-RADS for this target. With minimal fall-out and optimum sensitivity, we can see perfect outcomes.

## Figures and Tables

**Figure 1:** Conceptual diagram of presented growth region algorithm.

**Figure 2:** The diagram of the PNN method.

**Figure 3:** The diagram of the proposed model.

**Figure 4:** The results of the method provided for breast cancer detection.

**Figure 5:** Breast cancer detection. Top: input image; bottom: output image.

**Figure 6:** Results of the adaptive median filtration.

**Figure 7:** Results of the GMM method after filtration for a malignant tumor.

**Figure 8:** Results of the presented approach for a benign tumor.

**Figure 9:** Results of the presented approach for a normal breast.

**Figure 10:** The ROC curve of the presented method.

**Table 1:** Literature review summary.

	Authors	Method	Objective	Results
1	Ribli et al. [27]	Faster R–CNN used mammography to identify tumors and showed that this method was quite time-efficient; however, the faster R–CNN is generally weak, meaning that the training set must contain a large set of ROIs yet complete enough to include all possible waste changes	Diagnosis and classification of masses in breast tissue	The system can detect 90% of malignant lesions in the INbreast dataset with only 0.3 false-positive marks per image

2	Gao [28]	They used a low-energy image (LE) similar to full-field digital mammography (FFDM) and a recombination image; in the proposed algorithm, the shallow CNN has the task of “image reconstruction,” and the deep CNN has “extracting features”	Diagnosis and classification of masses in breast tissue	Experimental results on 89 FFDM datasets are obtained using recombinant “virtual” imaging features with an accuracy of 0.90 and AUC = 0.92

3	Jung et al. [29]	The model used a single-stage detector and a two-stage detector; one-step detectors such as RetinaNet generate a fixed number of projections over a network to cover possible positive sample spaces; unlike RetinaNet, the R–CNN mask can classify finite boxes in any range of scales and aspect ratios in any situation by segmenting the pixel surface	Diagnosis and classification of masses in breast tissue	The best result of this algorithm for TPR @ FPPI in the GURO dataset is (0.99 ± 0.01@3.0)
				(1.00 ± 0.00@1.3)
				(0.94 ± 0.03@0.5)

4	Shams et al. [30]	A deep generative multitasking network (DiaGRAM) has been used to solve data loss and limited training data to interpret the lesions because it is a costly and time-consuming task; this multifunctional network is built on a combination of Concentration neural networks and a generational opposite network	Classification of masses in breast tissue	The results of this algorithm for the INbreast dataset are as follows:
				Accuracy equal to 9.2% ± 5/93
				And AUC = 92.5 ± 2.4%

5	Al-masni et al. [31]	A CAD system based on deep learning ROI (area of interest) techniques using CNN called YOLO was developed to diagnose and classify breast masses into benign and malignant states in DDSM mammographic images	Diagnosis and classification of masses in breast tissue	The results of this algorithm are as follows
				Sensitivity = 93.2%
				Feature = 78%
				AUC = 87.7%

6	Chougrad et al. [32]	CAD describes a system based on deep CNN that distinguishes malignant and benign breast mass in high-resolution mammographic images; the models used are VGG16, ResNet50, and Inceptionv3	Classification of masses in breast tissue	With the ResNet50 network in the DDSM dataset, they achieved an accuracy of 27.27%

7	Ragab et al. [33]	The region-based method was used to determine the threshold of 76 and determine the most significant area; at the feature extraction stage, DCNN was used; AlexNet network retraining was used to distinguish between the two classes; for better accuracy, the last layer of DCNN was replaced with SVM	Diagnosis of masses in breast tissue	Accuracy, AUC, sensitivity, specificity, accuracy, and F1 score were 80.5%, 88.8%, 88.4%, 84.2%, 86%, and 81.5%, respectively

8	Hazarika and Mahanta [34]	The method of extraction of breast border area using threshold-based zoning with morphological operations was proposed; for this purpose, the two-stage image contrast enhancement method was used; in the first phase, a two-step histogram correction technique is used to improve the image at the general level, and in the second phase, a nonlinear filter based on local mean and the local standard deviation for each pixel is applied to the image with the modified histogram	Diagnosis of cancer in breast tissue	The result of the proposed algorithm with 322 images is 98% accuracy
9	Rajendra et al. [35]	Four texture extraction algorithms were used to extract features from mammographic images, and the SVM classification method was used to classify mammographic images into normal and abnormal categories	Classification of masses in breast tissue	The best results are related to the GLCM feature
				Accuracy = 92%, sensitivity = 94%, specificity = 93%, accuracy = 95%

10	Eltoukhy et al. [36]	The CAD system, based on feature extraction, was applied using the Gauss-Hermitage method, and the features were classified into four different categories: K-NN, random forest, and AdaBoost	Diagnosis of masses in breast tissue	The accuracy of the method used on the two sets of IRMA and MIAS images is 93.27 and 90.56, respectively

11	Padmavathy et al. [37]	A practical method was used by NSST + ANFIS to diagnose breast cancer; NSST was used to parse original images in multiple directions and several scales, and ANFIS-compliant clustering was used to classify input images	Diagnosis of masses in breast tissue	The results of the proposed algorithm
				Accuracy = 98.2%, sensitivity = 90.4%, specificity = 90.6%

12	Tahmooresi et al. [38]	A method for the early diagnosis of breast cancer has been proposed. In which it combines different machine learning methods, Support Vector Machine (SVM), ANN, KNN, Decision Tree (DT)	Classification of masses in breast tissue	Accuracy of 99.8% was achieved for the diagnosis of breast cancer

13	Amrane et al. [39]	They studied different machine learning methods such as support vector machine, Naive Bayes classifier, and nearest neighbor (KNN) to classify images of breast cancer and claimed that the KNN classification method performed better than vector machine; gain support and Naïve Bayes	Classification of masses in breast tissue	The KNN method has a higher accuracy of 97.57. However, the NB method also has a good accuracy of 96.99%

14	Anjaiah et al. [35]	Multi-ROI segmentation is one of the ways these authors have used mammography images; also, images were extracted using statistical criteria to measure the texture characteristics of mammographic images	Classification of masses in breast tissue	This method helps better detect the texture and shape of suspicious mammography images and better diagnose breast cancer

15	Vijayarajeswari et al. [40]	They efficiently categorized normal and abnormal classes into mammographic images using Huff transforms; improve results using other features such as mean, variance, and entropy; finally, the SVM cluster was used for classification	Classification of masses in breast tissue	The diagnosis accuracy in standard images is 65%, and in nonnormal images, 71%

16	Chowdhary et al. [41]	The goal of this study is to use intuitionistic possibilistic fuzzy c-mean clustering to segment medical photos	Segmentation of breast cancer	For MIAS pictures with varying noise levels of 5%, 7%, and 9% of the presented method, the average segmentation accuracy is 91.25 percent, 87.50 percent, and 85.30 percent

17	Chowdhary et al. [42]	Deep convolution neural networks are used to classify breast cancer using computer vision and image processing	Classification of breast cancer	For benign and malignant pictures, the traditional computer vision and image processing paradigm has a classification accuracy of 85 percent and 82 percent, respectively

**Table 2:** Comparison of the approach presented and selective seed methods from the approach to the growth area.

Method	Jaccard	Similarity
Growth region hand selection	0.82	0.63
Growth region FCM-GA selection	0.95	0.71
GMM method	0.93	0.65

**Table 3:** Comparison of the proposed algorithm with handy selection FCM-GA and GMM.

Method	RMS
Growth region hand selection	0.5711
Growth region FCM-GA selection	0.3681
GMM method	0.4216

**Table 4:** The results of performance analysis.

	Sensitivity	Specificity	Precision	Fall-out
Hand selection	0.72	0.65	0.76	0.35
FCM-GA selection	0.83	0.79	0.94	0.21
GMM method	0.76	0.63	0.92	0.37

**Table 5:** The results of detection parameters.

	Sensitivity	Specificity	Precision	Accuracy	Fall-out
MIAS	0.91	0.92	0.99	0.92	0.08
BI-RADS	0.88	0.72	0.95	0.80	0.28

## Data Availability

The mammography data of this study are available in the MIAS and BI-RADS repositories (the Mammographic Image Analysis Society Digital Mammogram Database, ACR BI-RADS® Mammography).
